This article has been retracted.

# Application of Image Processing Technology in Aerobics Injury Diagnosis

**DOI:** 10.1155/2022/2553048

**Published:** 2022-08-06

**Authors:** Duo Zhang, Yan Tian

**Affiliations:** ^1^Physical Education Department, Civil Aviation Flight University of China, Guanghan 618307, Sichuan, China; ^2^College of Physical Education, Chengdu University of TCM, Chengdu 611137, Sichuan, China

## Abstract

Aerobics sports injury diagnosis is a rapid diagnosis of sports injuries caused by athletes in the process of aerobics training or competition. The purpose of this paper is to use image processing technology to study and analyze the diagnosis of aerobics sports injury, so that the diagnosis results can be obtained more quickly and effectively. This paper first introduces the image processing technology and then analyzes the sports injury in colleges and universities. Firstly, the algorithm formula of image processing technology is given, and then the algorithm is introduced into the dynamic analysis of aerobics injury diagnosis. The two are compared through example analysis. The experimental results show that joint strain, sprains, and muscle strain are the main types of sports injury of College Aerobics students, reaching 59, 50, and 31 times, respectively. When using image processing technology in the diagnosis of sports injury, the diagnosis results can be obtained quickly and effectively.

## 1. Introduction

With the rapid development of image processing technology in China, we can find that it has been applied in various fields of real life. At the same time, image processing technology is also widely used in the detection of sports injuries. Most sports injuries can be diagnosed by image processing technology. Image processing technologies are a kind of using computers to deal with image messages. It primarily deals with image digitization, image intensification and repair, image data codes, image division, and image definition. Image processing technology has successfully entered people's lives and affected people's lives. And the image processing technology is excellent in the diagnosis of sports injury, especially in the diagnosis of aerobics sports injury.

Today, with the diversified and multiproject development of image processing technology, how to apply image processing technology perfectly in aerobics sports injury diagnosis and use image processing technology to obtain the best sports injury judgment also has far-reaching significance for the development and expansion of image processing technology. Image processing technology is also widely used. In recent years, scholars have used image processing technology to solve the problem of sports injury diagnosis, but there is relatively little application and research in aerobics sports injury diagnosis. How to reduce the occurrence of sports injuries in high-level competitive aerobics athletes is an important problem that needs to be solved urgently in the development of Chinese competitive aerobics. Therefore, the application of image processing technology to solve the problem of aerobics injury diagnosis has both theoretical and practical significance.

With the progress of society, increasing scholars have done relevant research on the application of image processing technology in aerobics injury diagnosis. In recent years, Wang J has normalized the image based on image recognition technology. And he carried out feature recognition on gray-scale images, ignoring small fluctuations. Combined with the characteristics of inventory images, he removed the drying process and proposed an algorithm model based on feature recognition [1]. However, the data used in his research is not the latest, and the results of the output are not very ideal. In the same year, Huang et al. studied the application of image processing technology in high-frequency vibration direction and amplitude measurement. According to the corresponding relationship between the vibration blurred images and the still images in the spectrum, they preprocessed the image [2]. However, their expressions on blurred images and still images were not clear enough. Before them, Oho E proposed an efficient and fast scanning method, such as TV scanning, combined with digital image processing technology to replace the traditional slow scanning mode as the standard acquisition model [3] of general scanning electron microscope (SEM). However, the combination of the two lacks theoretical support.

After studying the image processing technology of other scholars, Zhang D used the methods of literature, questionnaire, and mathematical statistics to investigate and analyze the common sports injuries of aerobics athletes. The results show that the common sports injury parts of aerobics athletes are waist, knee, shoulder, and ankle [4]. However, he did not make a systematic analysis of his research themes in the conclusion. Subsequently, Zhu et al. used big data analysis technology and computer vision technology based on convolutional neural network to establish the loss risk prediction model of aerobics athletes according to the relevant theories of sports biomechanics and computer image recognition [5]. However, the application effect of the prediction model created in real life is not very good. Later, Mmfa introduced the application of nuclear medicine technology in the diagnosis of bone and soft tissue injury, focusing on the important contribution of bone scintigraphy and hybrid research (SPECT/CT) [6]. However, his own arguments expressed in the article were relatively few, and most of them are a study of the research results of others. Unlike him, Jyoti et al. discussed a range of imaging options available in clinical settings for sports injuries and provided an in-depth understanding of the role of each imaging modality and image guidance procedure in enabling athletes to resume activities at an early stage [7]. Zhang observed and analyzed the effects of *Astragalus* and Salvia miltiorrhiza on skeletal muscle injury in aerobics athletes [8]. However, there is too much overlap in the methods he has used in his research.

The innovation of this paper lies in the following: (1) in the diagnosis of aerobics sports injury, it can use image processing technology to diagnose more quickly and effectively. It makes it easier for athletes to manage their physical condition. (2) Image processing technology algorithm is applied to the research of aerobics sports injury diagnosis. In other applications, image processing technology is often used as a method to check product quality problems. This paper is committed to deeply mining the internal characteristics and advantages of image processing technology and finds out the similarities between image processing technology and medical image diagnosis. It uses the characteristics of the algorithm to diagnose medical images to get a faster diagnosis result.

## 2. Application of Image Processing Technology in Aerobics Injury Diagnosis

### 2.1. Image Processing Technology

#### 2.1.1. Overview of Digital Image Processing

Digital image processing refers to a technology that takes corresponding operations on digital images with the help of computers to achieve the expected purpose, so we can also use the concept of computer image processing to represent digital image processing. Image is the representation of a natural landscape. It can be presented in various ways objectively. It includes visible images, such as light images, photos, graphics, and pictures. It also includes abstract mathematical functions and physical images that cannot be seen by human eyes [9]. From the perspective of whether the computer can recognize and process it, images can be divided into two categories. The first category is analog images, and the other category is digital images. Digital images are the research object of digital image processing technology.

#### 2.1.2. Content of Digital Image Processing

In real life, when processing digital images, if there is no other program to process the images directly, we will encounter many difficult places. For example, there is an interference signal in the image when the image is encoded and compressed. At this time, when we change the data of the original image into another way with obvious features, the image can be processed quickly and effectively. The most widely used image transformation methods are the following [10].

*(1) Fourier Transform*. Fourier transform is actually sending a signal from the time domain to the frequency domain, and the reciprocal of the time domain is its frequency. The speed of changing the gray level of an image is the frequency of the image.  Figure 1 shows the spectrum display of a medical image.

*(2) Wavelet Transform*. Wavelet transform is similar to Fourier transform. The function of wavelet transform is to send image data from the spatial domain to the wavelet domain. The wavelet coefficients obtained in this way are not single-layer, but multilayer. Wavelet transform is also a great tool for multilevel image decomposition. As shown in Figure 2, after the image is changed by wavelet, the subsequent work of the image is completed by reading and changing the wavelet coefficient. For example, changing the wavelet coefficient can change one aspect of the characteristics of the original image [11].

*(3) Main Contents of Image Processing Technology*. As shown in Figure 3, classic digital image processing mainly includes image enhancement, image transformation, image restoration, image edge detection, image segmentation, image feature parameter extraction, and image morphological processing, and the output is the processed image [12].

The main task of image analysis and recognition is to extract the features and measure the parameters of the target object obtained by image segmentation, to form the representation and description of non-images such as characters and values [13].

Image understanding is a kind of advanced digital image processing, which is a continuation and development of digital image processing and image analysis. It enables the computer to have the ability to understand the surrounding scenery like human beings, to replace human beings to solve practical application problems. After the operation of digital image understanding technology, the output is the description and interpretation of the image [14].

### 2.2. Image Preprocessing Algorithm

Image preprocessing is to transform the part image captured by the image acquisition device to achieve the purpose of image feature extraction and recognition. Many algorithms are involved in the process of image filtering, binarization, morphology, and edge detection. Therefore, the main research content of this chapter is to select suitable digital image processing methods and algorithms according to the actual characteristics of aerobics injury diagnosis [15].

#### 2.2.1. Filter Processing

The image captured by the camera may be disturbed by noise in the process of digitization, resulting in poor quality. Therefore, when further processing the digital image, it must be filtered first to eliminate or reduce the noise and restore the original image [16].

*(1) Mean Filtering*. It is a typical linear filtering algorithm. Its basic principle is to determine a template for the target image from the digital image. Its common template is square. Common 3 × 3 mean filtering 4-domain and 8-domain templates are shown as follows:

(1) $$\begin{array}{c} \frac{1}{5}\times \left[\begin{array}{ccc} 0 & 1 & 0\\ 1 & 1 & 1\\ 0 & 1 & 0 \end{array}\right]\frac{1}{9}\left[\begin{array}{ccc} 1 & 1 & 1\\ 1 & 1 & 1\\ 1 & 1 & 1 \end{array}\right]. \end{array}$$

*(2) Gaussian Filtering*. Gaussian filtering (also known as weighted filtering, it is also a kind of linear smoothing filtering) is suitable for eliminating Gaussian noise and is widely used in the noise reduction process of image processing [17]. Its function is expressed as

(2) $$\begin{array}{c} j\left(c,u\right)=\frac{1}{2\pi \sigma }r^{\left(c^{2}+u^{2}\right)/\left(2r^{2}\right)}. \end{array}$$

Among them, 2 *πσ* 2 represents the weighted average of the pixel values of the entire image, and the value of each pixel is obtained by the weighted average of its own value and other pixel values in the field. The commonly used templates for Gaussian filtering are similar to the mean template. The commonly used templates include 3 × 3 templates, 5 × 5 templates, and 7 × 7 templates. The commonly used 3 × 3 Gaussian template is shown as follows [18]:

(3) $$\begin{array}{c} \frac{1}{16}\times \left[\begin{array}{ccc} 1 & 2 & 1\\ 2 & 4 & 2\\ 1 & 2 & 1 \end{array}\right]. \end{array}$$

#### 2.2.2. Binarization Treatment

Image binarization processing is the basic technology of image preprocessing and a very active branch of image processing. Especially, it plays an important role in image information compression, edge extraction, and shape analysis. It has a wide range of applications and has become a basic segment in its processing process [19].

Binary image refers to the image with only two gray levels, which has small storage space and fast processing speed. It can conveniently carry out logical operation on the image [20]. After binarization, the image has only black and white, so the degree range is divided into target and background, and the binarization of the image is realized.

(4) $$\begin{array}{c} \left(h\left(c,u\right)\right)=\left\{\begin{array}{cc} 255\left(\text{white}\right) & g\left(c,u\right)\geq y\\ 0\left(\text{black}\right) & g\left(c,u\right)<y \end{array}\right.. \end{array}$$

#### 2.2.3. Global Threshold Method

In some simple images, the background region and the target region form two peaks in the histogram of the image, and a trough is formed between the two peaks [21]. Then, the gray value *y* represented by the trough between the two peaks is selected as the threshold to realize the segmentation of the two regions. This method is also known as the bimodal method, as shown in Figure 4.

If the image has 256 gray values, the gray value range is 0∼255, and then select a gray value y to divide the gray histogram into two categories *H*_0_ and *H*_1_. M represents the total number of image table points in the image, and *m*_*l*_ represents the number of image table points with gray value L [22]. Assuming that the number of pixels in *H*_0_ and *H*_1_ areas accounts for *e*_0_ and *e*_1_ in the overall image, and the average gray values of the two areas are *i*_0_ and *i*_1_, we can get the following:

Probability:

(5) $$\begin{array}{c} E_{0}=\overset{y}{\underset{l=0}{\sum }}q_{l}=\frac{\sum_{l=0}^{y}m_{l}}{M}, \end{array}$$

(6) $$\begin{array}{c} e_{1}=\sum_{l=k=1}^{n-1}q_{l}=1-e_{0}. \end{array}$$

Average gray value:

(7) $$\begin{array}{c} i_{0}=\sum_{l=0}^{k}lq_{l}, \end{array}$$

(8) $$\begin{array}{c} i_{1}=\sum_{l=y+1}^{n-1}lq_{l}. \end{array}$$

Then, the total average gray value:

(9) $$\begin{array}{c} i=e_{0}\times i_{0}+e_{1}\times i_{1}. \end{array}$$

Interclass variance:

(10) $$\begin{array}{c} h\left(y\right)=e_{0}\times {\left(i_{0}-i\right)}^{2}+e_{1}\times {\left(i_{1}-i\right)}^{2}=e_{0}e_{1}{\left(i_{0}-i_{1}\right)}^{2}. \end{array}$$

The optimal threshold is

(11) $$\begin{array}{c} Y=\text{ARGMAX}\left(H\left(Y\right)\right). \end{array}$$

#### 2.2.4. Maximum Entropy Threshold

According to the concept of entropy, for the image with a gray-scale range of 0, 1, 2,…, *N*−1, the entropy of the histogram is defined as

(12) $$\begin{array}{c} J=-\sum_{L=0}^{N-1}Q_{L}{\in \text{Q}}_{L}. \end{array}$$

*Q*_*L*_ is the probability of pixels with gray value *L* in the overall image. If the threshold *y* is set, the image is divided into target *P* and background *n*, and their probability distributions are as follows:

Zone *P*:

(13) $$\begin{array}{c} \frac{Q_{L}}{Q_{Y}}L=0,1,2,\ldots Y\;Q_{Y}=\sum_{L=0}^{Y}Q_{L}. \end{array}$$

Zone V:

(14) $$\begin{array}{c} \frac{Q_{L}}{1-Q_{Y}}L=Y+1,Y+2,\ldots ,N-1. \end{array}$$

If

(15) $$\begin{array}{c} J_{Y}=-\sum_{L=0}^{Y}Q_{L}{\in \text{Q}}_{L}, \end{array}$$

then it can get the following formula:

(16) $$\begin{array}{c} J\left(Y\right)=-\sum_{L=0}^{N-1}Q_{L}{\in \text{Q}}_{L}, \end{array}$$

(17) $$\begin{array}{c} J_{P}\left(Y\right)=-\sum_{L=0}^{Y}\frac{Q_{L}}{Q_{L}}\in \frac{Q_{L}}{Q_{L}}={\text{INQ}}_{Y}+\frac{J_{L}}{Q_{Y}}. \end{array}$$

Then, the total entropy of the image is

(18) $$\begin{array}{c} J_{N}\left(Y\right)=-\overset{N-1}{\underset{L=Y+1}{\sum }}\frac{Q_{L}}{1-Q_{Y}}\in \frac{Q_{L}}{1-Q_{Y}}=\text{IN}\left(1-Q_{Y}\right)+\frac{J-J_{Y}}{1-Y_{Y}}. \end{array}$$

#### 2.2.5. Principle of Mathematical Morphology

There are two basic operations in mathematical morphology: expansion and decay. Based on these basic operations, we can also deduce and combine various practical algorithms of mathematical morphology, such as open operations and closed operations.

*(1) Swell*. Image *s* is expanded with a structural element *n* and can be written as

(19) $$\begin{array}{c} S⊕N=\left\{C{|\left(\hat{N}\right)}_{C}\cap S\neq \emptyset \right\}. \end{array}$$

It first makes an image of the structural element *n* about its origin and then shifts the image *C* to the image *s*. Then, the set of elements formed when the image after translation intersects at least one nonzero common element of the target point in the image s is the result of the expansion operation. As shown in Figure 5, the shapes of structural elements can be rectangular, square, circular, diamond, and other shapes. In this example, only one structural element in rectangular form is selected.

*(2) Corrode*. The image *S* is etched by a structural element *N* to write *S*Θ*N*, which is defined as

(20) $$\begin{array}{c} S\Theta N=\left\{C{|\left(N\right)}_{C}\in S\right\}. \end{array}$$

When the structural element *N* is completely still contained in the image *S*, the set of the origin of the structural element *N* is the result of corrosion operation, as shown in Figure 6.

### 2.3. Aerobics Sports Injury

#### 2.3.1. Overview of Sports Injury

Some people say that the concept of sports injury is because external factors act on the human body, resulting in the normal operation of human organ function. It also causes discomfort in the human body, which is called injury. Similarly, we can know that the injury in sports is a sports injury. The injury caused by different sports has its remarkable characteristics, but one thing is common: the impact of sports injury on sports participants is extremely serious.

#### 2.3.2. Analysis on the Current Situation of Sports Injury of Aerobics Majors in Colleges and Universities

1. Through the survey, we can get Tables 1 and 2. Among the 160 students majoring in Aerobics selected by 8 colleges and universities in China, one male is an international athlete from Guangzhou Institute of Physical Education. There are 3 national athletes, 2 boys and 1 girl, from D University and a university, respectively. The proportion of students at the master level accounted for 2.49% of the respondents. The proportion of students at the national level and the national level is 8.13% and 20%, respectively. The proportion of students below national level II is the largest, 69.38%.
2. It can be seen that, with the continuous deepening of the training mode of sports talents combined with sports education in China, college students have also made good achievements in international Chinese competitions. However, it should also be noted that the number of students who have obtained the master level is small, accounting for only 2.49% of the selected research objects. From the perspective of gender, the number of girls majoring in aerobics is greater than that of boys, indicating that aerobics is more favored by girls.
3. Incidence and duration of sports injury: in the investigation on the incidence of sports injury of aerobics majors (Tables 3 and 4), we can see that there are many phenomena of sports injury of aerobics students during training. Among the 160 aerobics majors surveyed, 132 students have experienced sports injuries. Among them, the number of injured girls is more than that of boys. The incidence of sports injuries among students is 83%, which is quite amazing. Some students have sports injury accidents more than once, with a total of 186 injuries. In each stage of aerobics practice, no one was injured in the preparatory activities, which is related to the low intensity of preparatory activities. Sports injuries mostly occur in the process of difficult training, and 62 people's sports injuries occur in this practice stage. This shows that, with the continuous development of aerobics, the requirements for difficult movements are higher and higher, and the requirements for students' physical reserves are also higher and higher. This leads to the emergence of a series of sports injuries in the process of practicing difficult movements and complete sets of movements.
4. In the investigation of the occurrence time of sports *injuries*, it is found that aerobics majors in different regions have phased characteristics in the occurrence time of sports injury and show regional differences. As shown in Figure 7, in terms of time, October and December are the high incidence stage of sports injuries. During this period, 86 students majoring in aerobics had sports injuries, accounting for 46% of the total number of injuries.
5. Location and type of sports injury: through the *investigation* of the parts and types of sports injury of aerobics majors in colleges and universities, it is found that there are 8 easy parts of sports injury of aerobics majors in total. They are shoulder, elbow, wrist, waist, thigh, knee, calf, and ankle. Among the 186 cases of sports injury, the highest part of sports injury was the wrist, with 36 cases. The second is the knee joint with 32 people times, and the third is the ankle joint with 30 people times. Thighs, lower legs, waist, shoulders, and hips ranked fourth to eighth.
6. It is found from the survey results (as shown in Table 5) that joint strain, sprains, and muscle strain are several main types of sports injuries of college aerobics majors, reaching 59, 50, and 31 times, respectively. The prone parts of joint strain are the wrist, waist, and knee. This is related to the content and method of aerobics training. Sprains often occur in the ankle and knee.

## 3. Experiment and Application of Image Processing Technology in Aerobics Injury Diagnosis

### 3.1. Preprocessing of Aerobics Sports Injury Diagnosis Surface Image

The surface image of aerobics sports injury diagnosis is affected by image acquisition, image transmission, and on-site working environment, resulting in the reduction of the visual effect of the image, such as insufficient contrast, unclear image edge contours, noise in the image, image blur, and deformation, which will bring inconvenience to computer image processing and analysis. To enable the computer to analyze and process the image well, this paper first needs to preprocess the collected aerobics injury diagnosis surface image. Image enhancement is the basic content of digital image preprocessing, which lays a good foundation for subsequent image processing, especially image segmentation.

Image enhancement can enhance the contrast of the image and increase the difference between the target and the background. It removes the useless interference information in the image and enhances the target features in the image. The algorithms of image enhancement mainly include gray histogram enhancement, noise elimination, piecewise linear enhancement, Laplace operator, and various filtering methods. By using image enhancement technology, the quality of aerobics sports injury diagnosis images has been significantly improved. It improves the definition of aerobics injury diagnosis image and obtains good visual effect. It greatly reduces the influence of ambient noise on aerobics injury diagnosis image and reduces the difficulty of image segmentation in the next step.

#### 3.1.1. Gray Histogram

From the gray histogram of the image, we can get the gray range of the image, the distribution of gray level, and the average brightness of the whole image, so we can get the important basis for further image processing. In addition, the histogram represents the gray distribution of the object image, and the shape of this gray distribution will not scale with the rotation of the object. It will not even change due to external light. Therefore, to a certain extent, using the histogram of the object can effectively identify the object.

The surface histogram and equalization histogram of the aerobics injury diagnosis diagram are shown in Figure 8. It has been operated by the gray histogram of the original surface image of aerobics injury diagnosis, and the histogram corresponding to the gray image is obtained. It then performs histogram equalization on the gray histogram. It improves the quality of the image. The clarity, brightness, and contrast of the image have been enhanced, which provides convenience for subsequent image processing.

#### 3.1.2. Motion Injury Image Denoising

In the process of collecting and transmitting aerobics sports injury diagnosis images, it is affected by the industrial field environment, which will inevitably produce noise, resulting in some unknown black and white spots on the image. This not only affects the visual effect of the image, but also increases some interference information, which also leads to the decline of image quality. It is not conducive to the operation and processing of subsequent computers. To eliminate the interference of image noise, we need to study a suitable low-pass filter. It filters out the interference of high-frequency noise signal through low-pass filters, to achieve the purpose of removing noise, so the selection of low-pass filters is particularly critical. For noise removal, various filtering techniques can be used to remove noise, such as mean filter, median filter, and improved median filter. These technologies are based on low-pass filtering technology to achieve the effect of noise reduction.

This paper uses a median filter. Median filtering technology can not only reduce noise, but also preserve the contour of the original image to the greatest extent. The specific implementation is to sort the gray value of the pixel and the gray value of the pixels in the surrounding window for a point in the image disturbed by noise and the area centered on the point. The intermediate value is obtained to replace the original pixel value of a certain point, to neutralize the abrupt points in the image and achieve the purpose of image noise removal. The flow chart of the median filtering algorithm can be shown in Figure 9.

### 3.2. Segmentation of Aerobics Injury Diagnosis Image

The most basic function of image segmentation is to segment the image into target and background. The ultimate purpose of segmentation is to segment the required parts according to the application requirements and remove the useless information areas such as background. The basic image segmentation techniques include edge segmentation and threshold segmentation. These basic technologies can realize the binarization of images. However, according to different objectives, it combines different application requirements. When appropriate, it needs to take special image segmentation. Combined with the particularity of sports injury medical images, this topic adopts a special image segmentation technology, that is, the image segmentation algorithm based on mathematical morphology to realize the segmentation of sports injury medical images.

Generally speaking, it is necessary to carry out binary threshold segmentation on the preprocessed sports injury image. Through the binary threshold segmentation operation of the image, the gauze image is separated from the background, and then, with the help of the reconstruction technology in mathematical morphology, the features in the sports injury image are finally segmented and extracted. Through image segmentation, it provides an important basis for feature extraction of sports injuries. At the same time, it is also convenient for the subsequent analysis of the computer image processing systems. The quality of image segmentation seriously affects the result of feature parameter extraction and ultimately affects the accuracy of recognition and judgment of computer image processing system.

After binarization, all regions of the image are black except warp and weft, and the feature region we need to extract; that is, the target is in the black region. Therefore, it is necessary to reverse the image and convert the target of the defect area into a white image. The essence of image inversion is to perform nonoperation on each pixel value after binarization. The black-and-white conversion of the original binary image is realized through the operation of taking and repairing to analyze and process the target defects in the future.

Edges can be defined as the region with discontinuous gray change in the image. Image edge is the basis of image segmentation and feature parameter extraction. The edge detection algorithm can detect the gray discontinuous part and then extract the edge of the target image, which is convenient for the subsequent target segmentation. The common image edges are shown in Figure 10, from which we can see the type of gray mutation. To segment the edge of the image, we need to study the appropriate edge detector algorithm. Classical edge detection algorithms include Prewitt operator, Roberts operator, Sobel operator, Laplacian operator, LOG operator, and wavelet transform.

### 3.3. Feature Extraction and Aerobics Injury Diagnosis Map

In the previous chapters, we used a series of image preprocessing, image segmentation, and other technologies for the surface image of sports injury, which belong to the field of image processing. When processing the image of a sports injury diagnosis, what we send to the computer image processing system is the original digital image to be processed. After the application of a series of image processing algorithms in a computer image processing system, the output is still image. At this time, the image is a binary image, the amount of information of the image is greatly compressed, and the quality of the image has been significantly improved. Image preprocessing and image segmentation technology are ready for the analysis and recognition of defect images. The process of image analysis mainly includes image feature extraction and measurement of feature parameters, image classification, and feature judgment results. During image analysis, what we send to the computer is the segmented image of the sports injury surface. After the analysis and judgment of the image, it outputs the data information and representation of the feature rather than the image information. Finally, the surface feature detection system gives the judgment result. It mainly goes through three processes to complete the recognition and classification of sports injury surface images.

#### 3.3.1. Feature Extraction

To identify the types of sports injury images, feature extraction is needed first. In this paper, when extracting the features of sports injury images, the input is the binary image segmented by morphology. The output is the data of the motion injury image; that is, the motion defect image is described from another non-image field of view. It needs a process to make the computer have the ability to analyze and understand images like people. The first step is to measure the parameters of image features. The measured data also directly affect the result of image discrimination.

Feature extraction is the feature extraction and parameter measurement of the target object obtained by image segmentation to form a description of image data. This description is non-image, which can be character data or digital. The main extracted image features include edge features, gray features, texture features, and geometric features. The result of image feature extraction directly affects the accuracy of image analysis and recognition. If the method is not suitable, the image classification cannot be carried out. What kind of features are selected for the image and the parameter measurement of the selected features is the key to the accuracy of the detection results.

#### 3.3.2. Image Recognition

Generally speaking, image recognition is to recognize and classify images. The research of image recognition technology in this subject is to develop a sports injury feature detection system, which replaces manual automatic detection and recognition of surface features. The specific implementation process of sports injury recognition system is as follows: the first step is to collect the original sports injury image and convert the image information of the analog signal into digital image. It is then transmitted to the computer surface feature detection system for image processing. The second step is to preprocess the surface feature image of a sports injury, which can enhance the contrast between the image feature target and the background. It reduces the influence of noise on the image and improves the quality of the image. In the third step, firstly, the threshold segmentation algorithm is used to binarize the image, and then the main features such as broken hole, missing longitude, and broken weft are extracted from the background with the help of the segmentation method of mathematical morphology. The fourth step is the extraction of image features and the measurement of parameters. The focus of this step is to select effective features that can reflect the commonness and individuality of defects. The last step is to complete the identification and classification of aerobics injury diagnosis by using a certain discrimination principle through the extracted data information.

It is to automatically recognize the surface of the sports injury images and classify these surface features, which involves pattern recognition technology. Pattern recognition is a comprehensive application of a series of digital image processing algorithms. Through pattern recognition technology, the surface feature detection system can finally complete the recognition and classification of sports injury images. In fact, sports injury recognition is such a process: first, extract the geometric features of the image and measure the feature parameters, then classify and judge the sports injury image according to the designed classifier, and finally output the recognition results.

## 4. Discussion

This document is committed to the application research and design of image processing technology in the diagnosis of bodybuilding injury, and it is ideal for intricate analyzes and processing of bodybuilding injury diagnosis. It not only expands the scope of applying image processing technology, but also is a new venture to research the intricacies of diagnosing fitness injuries. Through the study of the process of image processing technology, this paper mines image processing technology as an important tool to study the complexity of the system. It holds great value in the study of the intricacy of injuries in exercise and health. In addition, based on the existing research of Chinese scholars, this paper draws on and summarizes it. The algorithm of image processing technology is listed one by one, making the algorithm suitable for the environment of sports injury medical images. For the research of image processing technology, this paper starts with the overview of the most basic image processing technology and analyzes the content and algorithm of the basic image processing technology. It was successfully combined and concluded with aerobic exercise injury diagnosis. In the empirical analysis stage, this paper uses the image preprocessing, segmentation and feature description algorithms listed in this paper to study the medical images of bodybuilding sports injury diagnosis. Several factors were analyzed, and the outcome indicates that the findings are in fact in line with the real world.

Discussion of the incident: it shows that image-based processing technology is more effective than a single observation of medical images. Athletes with sports injuries can judge the injury more quickly. This can greatly reduce the time to study sports injuries. In the specific practical decision-making, image processing technology can still analyze the medical image of sports injury and obtain the diagnosis results reasonably and flexibly, to obtain the most effective and rapid diagnosis.

This paper makes a case study on the medical image of aerobics injury diagnosis. Firstly, this paper makes a qualitative analysis of the concept and algorithms of image processing technology. Then, it studies the injury of aerobics athletes and uses the algorithm to combine and analyze according to the sports injury medical image. Through the analysis of the data, this paper concludes that the injury diagnosis of aerobics athletes based on image processing technology is indeed faster and more effective than human naked eyes.

## 5. Conclusion

Through the case study, this paper draws an important conclusion: through the application of image processing technology in aerobics sports injury diagnosis, we can find that using image processing technology can diagnose sports injury medical images more quickly. However, this is not absolute. It does not rule out the fixed nature of medical images. Some small details may not be seen by experienced doctors, such as the diagnosis of various injury degrees of Aerobics Athletes in this case. This requires more detailed research and quantitative analysis to determine a more effective diagnostic report. To reduce the injury rate of aerobics, it can reasonably supplement nutrition, adjust work and rest time, reduce exercise fatigue, do stretching and relaxation exercises, strengthen medical supervision and rehabilitation training, etc. The items discussed in this article are based on the combination of image processing technology and bodybuilding injury medical images, and the selection of items is relatively limited. The general reality of medical imaging of sports injuries will face more detailed diagnostic problems. In reality, aerobics injuries should also be studied in combination with many factors. If the study is more careful, it will be more valuable and more difficult. However, we can still choose to believe that there will be increasingly such research reports in the near future. And the image processing technology will be increasingly developed. Even subtle problems in medical images can be diagnosed in a short time.

## Figures and Tables

**Figure 1:** Medical image and its frequency domain spectrum display. (a) Medical image. (b) Frequency domain spectrum.

**Figure 2:** Binary wavelet decomposition of image.

**Figure 3:** Main content of image processing technology. (a) Schematic diagram of image processing. (b) Schematic diagram of image recognition. (c) Schematic diagram of image understanding.

**Figure 4:** Schematic diagram of bimodal method.

**Figure 5:** Schematic diagram of expansion.

**Figure 6:** Corrosion schematic diagram. (a) Image s. (b) Image n. (c) Image *S* Θ *N*.

**Figure 7:** time statistics of sports injury. (a) Time of sports injury. (b) Total damage of each month. (c) Percentage of damage at each time.

**Figure 8:** Gray histogram. (a) Histogram corresponding to the gray image. (b) Histogram homogenization effect.

**Figure 9:** Flowchart of median filtering algorithm.

**Figure 10:** Edge of image. (a) Stepped edge. (b) pulsed edge. (c) Stepped edge first-order difference. (d) Pulsed edge first-order difference. (e) Stepped edge difference. (f) Pulsed edge second-order difference.

**Table 1:** Sports grade of students majoring in aerobics.

	International master class	National elite level	The national level	National secondary	National level 2 or below	A combined
Male	1	2	9	33	33	65
Female	0	1	4	78	78	95
A combined	1	3	13	32	111	160
A combined%	0.63%	1.86%	8.13%	20%	69.38%	100%

**Table 2:** Regional distribution of sports grades of aerobics majors.

University name	International master class	National elite level	The national level	National secondary	National level 2 or below
A	0	2	3	9	6
B	0	0	2	4	14
C	0	0	0	6	14
D	1	1	5	8	5
E	0	0	0	1	19
F	0	0	3	4	13
G	0	0	0	0	20
H	0	0	0	0	20
A combined	1	3	13	32	111

**Table 3:** Incidence of sports injury in aerobics majors.

	The number of survey	The number of injured	Incidence of injury (%)	The number of injured	Average number of injured
Male	64	51	78	97	1.48
Female	96	81	87	172	2.66
A combined	160	132	84	186	1.16

**Table 4:** Exercise period of sports injury of aerobics majors.

	Preparation activities	Difficulty movement training	Flexible training	Complete set of training	Strength training
Male	0	20	13	12	5
Female	0	42	10	15	15
A combined	0	62	23	27	20

**Table 5:** Parts and types of sports injury of aerobics majors.

	Joint sprains	Strain	Strain	A cramp	Contusion	Scratch	Fractures	A combined
The head								
The shoulder	6	3						9
The elbow					6	2	2	8
Wrist			34		2			36
The waist	5		10					15
Thighs, hips		28						28
The knee joint	9		15			8		32
Ankle	30							30
The calf				20		8		28
A combined	50	31	59	20	8	16	2	186

## Data Availability

The data underlying the results presented in the study are available within the manuscript.
